The article "A Framework on Performance Analysis of Mathematical Model-Based Classifiers in Detection of Epileptic Seizure from EEG Signals with Efficient Feature Selection" was published in 2022. Journal: J Healthc Eng.

# A Framework on Performance Analysis of Mathematical Model-Based Classifiers in Detection of Epileptic Seizure from EEG Signals with Efficient Feature Selection

**DOI:** 10.1155/2022/7654666

**Published:** 2022-09-06

**Authors:** V. S. Hemachandira, R. Viswanathan

**Affiliations:** Department of Mathematics, Kongu Engineering College, Perundurai, Erode 638060, Tamil Nadu, India

## Abstract

Epilepsy is one of the neurological conditions that are diagnosed in the vast majority of patients. Electroencephalography (EEG) readings are the primary tool that is used in the process of diagnosing and analyzing epilepsy. The epileptic EEG data display the electrical activity of the neurons and provide a significant amount of knowledge on pathology and physiology. As a result of the significant amount of time that this method requires, several automated classification methods have been developed. In this paper, three wavelets such as Haar, dB4, and Sym 8 are employed to extract the features from A–E sets of the Bonn epilepsy dataset. To select the best features of epileptic seizures, a Particle Swarm Optimization (PSO) technique is applied. The extracted features are further classified using seven classifiers like linear regression, nonlinear regression, Gaussian Mixture Modeling (GMM), K-Nearest Neighbor (KNN), Support Vector Machine (SVM-linear), SVM (polynomial), and SVM Radial Basis Function (RBF). Classifier performances are analyzed through the benchmark parameters, such as sensitivity, specificity, accuracy, F1 Score, error rate, and g-means. The SVM classifier with RBF kernel in sym 8 wavelet features with PSO feature selection method attains a higher accuracy rate of 98% with an error rate of 2%. This classifier outperforms all other classifiers.

## 1. Introduction

Epilepsy is an immensely sensitive and intensely fatal neurological disorder. Approximately, 1% of the world population is suffering from this ailment. It is normally identified by analyzing EEG signals [1]. In the clinics, visual observation of EEG signals is leaned on as the standard method to detect it. This type of detection is time-consuming and induces a lot of errors. Above all, the epileptic seizure should be timely and accurately diagnosed before the patient goes to an ictal state [2]. Hence, an accurate seizure detection system will serve as a top-of-the-line boon to humanity. Various methods of seizure detection technique have been attended; these methods are broadly classified into three major groups: Feature extraction techniques, feature selection, and classifiers [3]. The interpretation and identification of epilepsy using EEG signals have emerged as an interesting study field in the last a few decades. Identification of epileptic seizures, spike detection, interictal and ictal analysis, linear and nonlinear analysis, and optimization algorithms have all been extensively studied [4].

The article "A Framework on Performance Analysis of Mathematical Model-Based Classifiers in Detection of Epileptic Seizure from EEG Signals with Efficient Feature Selection" was published in 2022. Journal: J Healthc Eng.

Epilepsy is characterized by abrupt disturbances in the brain's electrical activity, and it is a condition that afflicts a significant number of individuals all over the globe. Epilepsy can lead to many serious injuries, such as broken bones, accidents, and burns. Some of these injuries could even be fatal. This issue reflects a very high societal cost for families of the middle class, and as a result, it causes a great deal of financial difficulties for such families. Both surgical and pharmaceutical approaches may be used, depending on the patient's epilepsy degree of severity, in order to successfully treat the condition [3]. It is not possible to properly manage seizures in all people by using antiepileptic medication, and surgery may also not be an option for certain patients due to the severity of their condition [4].

Therefore, forecasting the onset of an epileptic seizure and then identifying the kind of seizure that has occurred is highly significant. The technique for feature extraction, feature selection, and classification is explained in tremendous detail in this article. There are significant number of publications that have been presented in the literature about the identification of epilepsy based on EEG data.

### 1.1. Related Works

Discrete wavelet transform (Haar, dB4, Sym8) was employed to extract EEG signal features, and epilepsy risk levels were identified using EM, MEM, and SVD classifiers with code converter technique by Harikumar et al. [4] with an overall accuracy of 97.03% achieved. Murugavel and Ramakrishnan [5] utilized the wavelet transform with approximate entropy to extract the features of EEG signals and multiclass SVM with ELM to identify the epilepsy seizures and reached 96% of classification accuracy. Truong et al. [6] described a hills algorithm to extract the EEG features with a sensitivity of 91.95% and a specificity of 94.05%, and their data demonstrated the efficacy of their proposed approach. Manjusha and Harikumar [7] proposed detrend fluctuation analysis with power spectral density to reduce the dimensionality of EEG data. K-means clustering and KNN classifier were applied to identify the epilepsy risk levels. The proposed work achieved 90.48% of sensitivity and 92.85% of specificity. Radüntz et al. [8] projected a support vector machine (SVM) and artificial neural network (ANN) to identify the epilepsy risk levels, and they used two classification methods, SVM and ANN, and found that ANN was more accurate than SVM (95.85% vs. 94.04%).

The article "A Framework on Performance Analysis of Mathematical Model-Based Classifiers in Detection of Epileptic Seizure from EEG Signals with Efficient Feature Selection" was published in 2022. Journal: J Healthc Eng.

Ijaz et al. [9] utilized hybrid prediction model with density-based spatial clustering of applications with noise to detect the outliers of diabetes and hypertensions data and synthetic minority over sampling technique with random forest to identify the diabetes and hypertensions and reached 92.56% of classification accuracy. Vulli et al. proposed a fast AI and a one-cycle policy with tuned dense net 169 to normalize the breast data. The proposed model was used to detect breast cancer metastasis. The proposed work achieved 97.4% accuracy [10]. Ghaemi et al. [11] utilized the improved binary gravitation search algorithm with wavelet domain to extract the features of EEG signals and SVM to identify the optimal channels and reached 80% of classification accuracy. Binary particle swarm optimization (BPSO) was used to choose the best channels, and Gonzalez et al. [12] used fisher discriminant analysis to find the auditory event-related potentials, which gave the best accuracy overall. Poli [13] analyzed the applications of particle swarm optimization (PSO). Independent component analysis (ICA) was employed to extract EMG signal features, and muscle activation intervals were identified using wavelet transform by Azzerboni et al. [14]. Greco et al. [15] used ICA to minimize EMG signal interference and the Morlet wavelet transform to determine muscle activation intervals. To detect the features of an epileptic seizure, various expansion methods have been proposed in the literature, such as discrete wavelet transform (DWT), continuous wavelet transform (CWT), Fourier transform (FT), discrete Fourier transform (DFT), fast Fourier transform (FFT), and short-term Fourier transform (STFT). From the detailed literature survey, it is acceptably assumed that DWT is the best method to detect seizure features. The DWT has the advantage of evaluating the signal in both the time and frequency domain. The following is the list of most important objectives that this research aims to achieve:

- In DWT, Haar, db4, and Sym8 techniques are proposed in this study to detect the seizure feature.
- Besides, this research proposes the Particle Swarm Optimization technique to select the best feature.
- The derived features from DWT are fed into the classifier for further classification. Normally classifiers are used to identify the signals, whether it has epileptic or not. The seven classifiers LR, NLR, GMM, K-NN, and SVM (Linear, Polynomial, and RBF) are used in this study.

The organization of the paper is as follows: Section 2 describes the materials and methods and explains the Haar wavelet, dB4 wavelet, and Sym8 wavelet-based feature extraction of EEG signals, Section 3 discusses the PSO-based feature selection, Section 4 describes the Classifiers, Section 5 exhibits results and discussion and Section 6 presents the conclusion and future work.

The article "A Framework on Performance Analysis of Mathematical Model-Based Classifiers in Detection of Epileptic Seizure from EEG Signals with Efficient Feature Selection" was published in 2022. Journal: J Healthc Eng.

## 2. Materials and Methods

The suggested method for automated epileptic seizure detection is presented in this section. The schematic diagram of the proposed method is shown in Figure 1. In this schematic diagram, the effectiveness of the EEG signal is maximized in the feature extraction stage by using multiple feature extraction approaches. The remainder of this section provides a full discussion of the feature extraction techniques used. A Particle Swarm Optimization (PSO) technique is used to choose the best features of epileptic seizures after the features have been extracted. After feature extraction and selection, the extracted and selected features are deployed to several classifiers, and performance benchmark results are analyzed and compared. The most effective classifiers have the highest benchmark value. Next, the dataset and specifics of each subsystem are detailed. The implementation environment details of the study are given in Table 1.

As given by Table 1, all of the datasets from A to E have 100 epochs. There are 4096 EEG sample values recorded throughout each epoch. The input EEG signals of [4096 × 100] samples per set are reduced to [256 × 100] estimated sample values after passing through wavelets at level 4 decomposition. The input EEG signals of [256 × 100] samples per set are again scale down to [256 × 10] estimated sample values after passing through PSO feature selection. The MATLAB 2019a environment was utilized for each and every simulation that was executed.

### 2.1. Data Description

The publicly available Bonn University datasets are chosen for the analysis. The Bonn University EEG datasets have A, B, C, D, and E with a sampling frequency of 173.6 Hz [16]. Dataset A represents the normal signal, and E represents the abnormal (epileptic seizure) signal, which is considered for this analysis. The details of the dataset are exhibited in Table 2. All of these segments have 100 epochs, with a recording period of 23.6 seconds. In sets (A) and (B), signals were obtained from healthy patients who would not even have epilepsy, with the set (A) being recorded when the subjects' eyes were open and set (B) when their eyes were closed. Signals from patients with epilepsy were obtained in sets (C), (D), and (E). For set (C) and (D), signals were composed of epileptic patients but not during an incidence of epilepsy, whereas in Set (E), signals were obtained from individuals during an existence of epilepsy [17]. Each epoch has 4096 samples of EEG signal. In this research, we purport to perform the analysis on the A–E epilepsy sets only.

The article "A Framework on Performance Analysis of Mathematical Model-Based Classifiers in Detection of Epileptic Seizure from EEG Signals with Efficient Feature Selection" was published in 2022. Journal: J Healthc Eng.

### 2.2. Wavelet Feature Extraction

In this work, the first step in analyzing epileptic seizures is the extraction of features from the obtained EEG datasets from the Bonn University database. Discrete wavelet transform (DWT) is used to extract the EEG features. The three wavelet families employed for feature extraction from EEG signal (A-E Bonn) datasets at level 4 wavelets decomposition are Haar wavelet (HAAR), dB4 wavelet (Daubechies), and Sym8 wavelet (Symlet8). After passing through the wavelets at level 4 decomposition, the input EEG signals of [4096 × 100] samples per set are reduced to [256 × 100] approximate values of samples. The essential features of wavelets are described in the following section of the paper.

#### 2.2.1. Haar Wavelet

It is essentially a discontinuous function that appears like a step function. It is a wavelet that is comparable to Daubechies dB1. The Haar wavelet is a basic kind of compression that involves average and difference terms, storing detail coefficients, removing data, and reconstructing the matrix to make it seem like the original matrix [18]. Only the Haar wavelet is well supported, orthogonal, and symmetric. The Haar decomposition has excellent time localization because of the compact support of the Haar wavelets [19]. The mathematical expression of the Haar wavelet function (*ψ*_*j*,*k*_) and scaling function (*ø*_*j*,*k*_) is represented as follows:

(1) $$\begin{array}{c} \psi_{j,k}\left(x,y\right)=\left\{\begin{array}{c} x+\pi ,-\pi \leq x\leq \frac{-\pi }{2}\\ \frac{\pi }{2},\frac{-\pi }{2}\leq x\leq \frac{\pi }{2}\\ x-\pi ,\frac{\pi }{2}\leq x\leq \pi \end{array}\right)\text{,}\\ {ø}_{j,k}\left(x,y\right)=f\left(x\right)=\left\{\begin{array}{c} 1,0\leq x\leq 1\\ 0,otherwise \end{array}\right)\text{.} \end{array}$$

#### 2.2.2. dB4 Wavelet

Ingrid Daubechies, one of the most lustrous luminaries in the domain of wavelet research, devised compactly supported orthonormal wavelets, which made discrete wavelet analysis feasible. The order of the Daubechies family wavelets is *N*, and dB is the wavelet's “family name.” These wavelets are energy-saving since they are orthogonal and compactly supported [20]. dB4 wavelet function is utilized in this work. Due to the overlapping windows used by Daubechies (dB) wavelets, all high-frequency changes are reflected in the spectrum of the high-frequency coefficient. Filter coefficients are used to create the Daubechies (dB) family of wavelets and scaling functions [21]. The 2*π* cyclic trigonometric polynomial related with the filter {*h*_*k*_} is the first step in Daubechies technique to creating orthogonal compactly supported wavelets. The filter's element sequence is deduced as follows [22]:

(2) $$\begin{array}{c} h_{k}=\int \emptyset \left(x\right)\sqrt{2}\emptyset \left(2x-k\right)dx. \end{array}$$

The mathematical expression of the Haar wavelet scaling function (*m*_0_(*ω*)) is represented as

(3) $$\begin{array}{c} m_{0}\left(\omega \right)=\frac{1}{\sqrt{2}}\underset{k\in Z}{\sum }h_{k}e^{-ik\omega }\text{.} \end{array}$$

By creating this function to provide orthogonally and smoothness, a new family of wavelets may be generated. As dB4 has a very small basis function, it may separate signal discontinuities more effectively.

The article "A Framework on Performance Analysis of Mathematical Model-Based Classifiers in Detection of Epileptic Seizure from EEG Signals with Efficient Feature Selection" was published in 2022. Journal: J Healthc Eng.

#### 2.2.3. Sym8 Wavelet

The Symlet wavelet family is an abbreviation for “symmetrical wavelets.” They are well constructed also to have the least amount of asymmetry and the greatest number of vanishing moments for a certain compact support. In this work, a wavelet function of type Sym8 was used. Sym8 Wavelet is a nearly symmetrical and smooth wavelet function [23]. In order to identify the presence of nonlinearity in the wavelet features, the statistical parameters, such as Mean, Variance, Skewness, Kurtosis, Pearson correlation coefficient, Canonical Correlation Analysis (CCA) for without feature selection method are given in Table 3.

As indicated in Table 3, the statistical parameters of the wavelet feature depict the presence of nonlinearity among the A–E sets for all three wavelets. Pearson Correlation Coefficient (PCC) exhibits peculiar types of no correlation in the intra epochs of A set. At the same time, CCA demonstrates more correlation among the two classes of A–E sets. This is an indication that features in the A–E sets are correlated and overlapped. It glitters in the histogram plots shown below.

Histogram of Haar Wavelet features for Epilepsy E-Set is exposed in Figures 2 and 3 displays the Histogram of Haar Wavelet features for Normal A-Set.  Figure 2 demonstrates the nonlinear nature of the wavelet features of the E-set with less outlier.  Figure 3 flaunts the availability of outlier in the wavelet features for normal A-set. Finally, these extracted features are then fed as input to the feature selection using Particle Swarm Optimization (PSO) algorithm.

## 3. PSO as a Feature Selection Algorithm

PSO is an illustrious method developed by Kennedy and Eberhart in 1995 [24]. Each search space is traversed by a collection of particles. The parameters for location *y* and velocity *w* are included in each swarm member *i*. Each particle's location parades a possible optimization solution.

### 3.1. Algorithm for PSO

Consider an N-dimensional space with *N* particles, each of which represents a significant solution. Particles then are propelled into hyperspace, where their positions are influenced by their own and neighbors' experiences. Each and every particle is represented as a potential solution to the obvious problem in a *D*-dimensional space in the basic formulation of PSO [25]. In a *D*-dimensional space, the particle *i* is represented as follows:

(4) $$\begin{array}{c} Y_{i}=\left(y_{i1},y_{i2},y_{i3},\ldots ,y_{iD}\right). \end{array}$$

Furthermore, each particle remembers its prior optimum location. The *i*^*th*^particle's best prior location may be expressed as

(5) $$\begin{array}{c} P_{i}=\left(p_{i1},p_{i2},p_{i3},\ldots ,p_{iD}\right). \end{array}$$

The *i*^*th*^ particle's velocity is expressed as follows:

(6) $$\begin{array}{c} V_{i}=\left(v_{i1},v_{i2},v_{i3},\ldots ,v_{iD}\right)\text{.} \end{array}$$

The greatest fitness value is assigned to the global best. The best particle in the world is chosen from all the particles in the population. It is mathematically expressed as follows:

(7) $$\begin{array}{c} P_{g}=\left(p_{g1},p_{g2},p_{g3},\ldots ,p_{gD}\right)\text{.} \end{array}$$

The cognitive component represents the location of the velocity adjustments made by the particle's prior best position. In contrast, the social component represents the position of the velocity adjustments made by the particle's global best position and is expressed as follows [26].

(8) $$\begin{array}{c} \left.W_{i}\left(k+l\right)=wV_{i}\left(k\right)+\eta 1\;r1\left(k\right)*\left(P_{i}\right.\left(k\right)-Y_{i}\left(k\right)+\eta 2\;r2\left(k\right)*\left(s_{i}\right.\left(k\right)*\;\left(s_{i}\right.\left(k\right)-Y_{i}\left(k\right)\right),\\ y_{i}d\left(t+1\right)=y_{i}d\left(t\right)+v_{i}d\left(t\right), \end{array}$$

where *w* denotes the inertia weight, *η*1 and *η*2 represent the positive acceleration constants. The velocity vector drives the optimization process, which in turn depicts the socially exchanged information.  Figure 4 determines the performance of MSE in a number of iteration for PSO feature selection at different weights. It is observed from Figure 4 that the optimum weight is chosen at = 0.5 with lower MSE values compared with other weights values. In this circumstance, inertia (*w*) is set to 0.5, while *η*1 and *η*2 are both set to 1. The output of PSO feature selection will make [256 × 100] input as wavelet features are reduced to [256 × 10].

The article "A Framework on Performance Analysis of Mathematical Model-Based Classifiers in Detection of Epileptic Seizure from EEG Signals with Efficient Feature Selection" was published in 2022. Journal: J Healthc Eng.

Let us, forthwith, analyze the presence of nonlinearity in the PSO features. In this case, the statistical parameters, such as Mean, Variance, Skewness, Kurtosis, Pearson correlation coefficient, and Canonical Correlation Analysis (CCA) are the best-suited ones. Hence, these parameters are extracted with wavelet feature along with the PSO feature selection method, and the same is given in Table 4. From Table 4, the statistical parameters indicate the presence of nonlinearity for the PSO features among both classes. PCC demonstrates the uncorrelated condition among the intraclass PSO features among the classes. CCA also distinguishes the noncorrelation among inter-classes that are A–E sets.

The normal probability plot for dB4 wavelet coefficient with PSO feature selection for Epilepsy E-Set is shown in Figures 5 and 6 displays the normal probability plot for dB4 wavelet features with PSO feature selection for Normal A-Set. It is observed from Figures 5 and 6 that the PSO features for dB4 wavelet feature extraction exhibits uncorrelated, overlapped, and nonlinear nature of the A–E sets.

The extracted features without PSO feature selection and with PSO feature selection are then fed as input to the various classifiers like linear regression (LR), nonlinear regression (NLR), Gaussian mixture model (GMM), K-Nearest Neighborhood (K-NN), SVM (Linear), SVM (Polynomial), and SVM (RBF) classifiers. These are discussed in the following sections.

## 4. Mathematical Model-Based Classifiers for Epilepsy Detection

In this section, model-based classifiers are used to classify the features that were extracted and selected with the help of wavelet (Haar, db4, and sym8) techniques and PSO methodology.

### 4.1. Linear Regression

Linear regression is a supervised learning technique in which one or more independent variables are linearly connected to the dependent variable [27]. Simple linear regressions employ only one independent variable, whereas multiple linear regressions use several independent variables [28]. A residue value is computed depending on the targeted value using conventional linear regression. The linear regression model equation is then implemented to the residue value. The performance of the classifier is evaluated based on the variation from its target value. Mathematical expression for simple linear regression is as follows:

(9) $$\begin{array}{c} Y=a+bX, \end{array}$$

where *Y* represents the dependent variable(*y* − *axis*), *X* represents the independent variable(*X* − *axis*), *b* indicates the slope line, and *a* represents the intercept of*y*. Therefore, slope line (*b*) and intercept (*a*) mathematically expressed as follows:

(10) $$\begin{array}{c} a=\frac{\left(\sum y\right)\left(\sum x^{2}\right)-\left(\sum x\right)\left(\sum xy\right)}{n\left(\sum x^{2}\right)-{\left(\sum x\right)}^{2}},\\ b=\frac{n\left(\sum xy\right)-\left(\sum x\right)\left(\sum y\right)}{n\left(\sum x^{2}\right)-{\left(\sum x\right)}^{2}}. \end{array}$$

The article "A Framework on Performance Analysis of Mathematical Model-Based Classifiers in Detection of Epileptic Seizure from EEG Signals with Efficient Feature Selection" was published in 2022. Journal: J Healthc Eng.

### 4.2. Nonlinear Regression

Nonlinear regression (NLR) is a regression analysis method in which empirical data are represented by a function that depends on one or more independent variables and is a nonlinear combination of model parameters. An approach of successive approximations is used to fit the data. Statistical model for nonlinear regression is expressed as follows [29]:

(11) $$\begin{array}{c} y∼f\left(x,\beta \right), \end{array}$$

where *x* represents the independent variables of vector, *y* indicates the dependent variables of vector, and *f* represents the expectation nonlinear function. Thereupon, expectation nonlinear function *f* mathematically is expressed as follows:

(12) $$\begin{array}{c} f\left(x,\beta \right)=\frac{\beta_{1}x}{\beta_{2}+x}. \end{array}$$

On the basis of the target set, a residue value is computed. The performance is then evaluated by applying the residue value and the EEG signal samples to the nonlinear equation.

### 4.3. Gaussian Mixture Model (GMM)

The Gaussian mixture model (GMM) is a weighted sum of Gaussian component densities that defines a parametric probability density function. Arbitrary density modeling is possible with GMMs with numerous coefficients. The random vector with probability density is expressed as follows [30]:

(13) $$\begin{array}{c} a\left(x\right)=\overset{L}{\underset{z=1}{\sum }}B_{i}\emptyset \left(a|C_{i},D_{i}\right)\text{,} \end{array}$$

where *L* represents the number of Gaussian mixture components, *B*_*i*_indicates the weight of the mixture. Therefore, the mixing parameters (*θ*) are often computed by increasing the log-likelihood function. Mathematical expression for log-likelihood function as follows:

(14) $$\begin{array}{c} F\left(\theta \right)=\overset{M}{\underset{y=1}{\sum }}\ln\left[\overset{L}{\underset{z=1}{\sum }}B_{i}\emptyset \left(a|C_{i},D_{i}\right)\right]. \end{array}$$

The expectation-maximization (EM) method is a frequently employed strategy for maximum likelihood outcomes.

### 4.4. K-Nearest Neighborhood (K-NN)

The K-nearest neighborhood (K-NN) method is based on the supervised learning approach and is one of the most basic machine learning algorithms. The K-NN approach may be wielded for both regression and classification. However, it is more commonly utilized for classification tasks [31]. The steps of the K-NN algorithm are as follows:

  Step 1: choose a neighbors' number *K*
  Step 2: determine the Euclidean distance between *K* neighbors
  Step 3: using the estimated Euclidean distance, find the *K* closest neighbors
  Step 4: compute how many data points each category has between all these *K* neighbors
  Step 5: define the additional data points to the class with the highest number of neighbors

The article "A Framework on Performance Analysis of Mathematical Model-Based Classifiers in Detection of Epileptic Seizure from EEG Signals with Efficient Feature Selection" was published in 2022. Journal: J Healthc Eng.

### 4.5. Support Vector Machine (SVM)

SVM is widely used for pattern classification. The SVM algorithm is applied to separate nonlinear samples into another higher dimensional space by kernel functions and then to locate the optimal separating hyperplane by solving a quadrate optimization problem [32]. The kernel function of SVM is the linear kernel, polynomial kernel, radial basis function (RBF), and sigmoidal neural network kernel. SVM–Linear, SVM-RBF, and SVM-Polynomial are used in this work.

(15) $$\begin{array}{c} Linear\;SVM:k\left(x,x_{i\;}\right)=x_{i\;}^{T}x,\\ Polynomial\;kernel\;of\;degree\;2:k\left(x,x_{i\;}\right)={\left(1+x_{i\;}^{T}x\right)}^{2},\\ RBF\;SVM\;:k\left(x,x_{i\;}\right)=\frac{\exp\;\left(-\gamma {\left\|x-x_{i}\right\|}^{2}\right)}{2\sigma^{2}}, \end{array}$$

where *γ* represents the bandwidth of the kernel and *σ* indicates the positive parameters to standardize the radius.

## 5. Results and Discussion

This paper considers regular 10-fold training and testing with 90% and 10% of the input features used for training and testing, respectively [33]. Table 3 highlights the average MSE results for Haar, dB4, and Sym8 wavelet features in various classifiers without PSO feature selection, and Table 5 illustrates the Average MSE for Haar, dB4, and Sym8 wavelet features in various classifiers with PSO feature selection.  Table 6 depicts the confusion matrix for the seizure detection.  Table 7 displays the Average performance of the classifier for Haar, dB4, and Sym8 wavelet features in various classifiers without PSO feature selection, and Table 8 exhibits the average performance of classifier for Haar, dB4, and Sym8 wavelet features in various classifiers with PSO feature selection. The following performance parameter measurements may be calculated and employed to examine the classifier's performance based on the confusion matrix. The following are the formulae for the sensitivity, specificity, accuracy, F1 Score, error rate, and *G*-mean and MSE.

From Table 6, True-Positive is represented as TP, True-Negative as TN, False-Positive as FP, and False-Negative as FN [34]. A TP states a positive sample that has been accurately forecasted as positive. A TN states a negative sample that has been accurately forecasted as negative. A FP occurs when a result is incorrectly assumed to be positive but is really negative. A FN occurs when a result is incorrectly assumed to be negative when it is really positive [35].

The Sensitivity is computed as follows:

(16) $$\begin{array}{c} Senstivity=\frac{TP}{TP+FN}*100\text{.} \end{array}$$

The specificity is expressed as follows:

(17) $$\begin{array}{c} Specificity=\frac{TN}{TN+FP}*100. \end{array}$$

The overall accuracy of the classifier is computed as follows:

(18) $$\begin{array}{c} Accuracy=\frac{TN+TP}{TN+TP+FN+FP}*100\text{.} \end{array}$$

F1 Score is expressed as follows:

(19) $$\begin{array}{c} F1\;score=\frac{2TP}{2TP+FP+FN}*100\text{.} \end{array}$$

Geometric Mean (G-mean) is computed as follows:

(20) $$\begin{array}{c} G-mean=\sqrt{\frac{TP}{TP+FN}*\frac{TN}{TN+FP}}. \end{array}$$

Mean Square Error (MSE) is computed as follows [36]:

(21) $$\begin{array}{c} MSE=\frac{1}{B}\overset{B}{\underset{i=1}{\sum }}{\left(P_{i}-Q_{j}\right)}^{2}\text{,} \end{array}$$

where *P*_*i*_ indicates the value of observed at a particular time, *Q*_*j*_ represents the value of target at typical*j*(*j* = 1 *to* 100), and *B* represents the number of observations per patient, in our case, which is 25600.

The article "A Framework on Performance Analysis of Mathematical Model-Based Classifiers in Detection of Epileptic Seizure from EEG Signals with Efficient Feature Selection" was published in 2022. Journal: J Healthc Eng.

Table 7 shows the average MSE for Haar, dB4, and Sym 8 wavelet features in various classifiers without feature selection. From Table 7, it is observed that for the Haar wavelet, SVM with RBF kernel classifier attains a low MSE value of 2.14*E* − 05. In the case of the dB4 wavelet, the GMM model achieves a low MSE value of 2.98*E* − 05, For Sym 8 wavelet; once again SVM(RBF) classifier reaches the top with a low MSE value of 8.89*E* − 06. The low value of MSE always demonstrates higher classification accuracy of the Classifier.

Table 8 depicts the average MSE for Haar, dB4, and Sym 8 wavelet features in various classifiers with the PSO feature selection method. Table 8 depicts that Haar wavelet SVM with RBF kernel classifier attains a low MSE value of 3.48*E* − 06. In the case of the dB4 wavelet, the KNN model achieves a low MSE value of 7.44*E* − 06. For Sym 8 wavelet, the SVM(RBF) classifier reaches the top with a low MSE value of **1.96*E* − 06**. The low value of MSE always demonstrates higher classification benchmark parameters of the Classifier.

Table 9 portrays the average performance measures like Sensitivity, Specificity, Accuracy, F1 Score, Error Rate, and G-mean for Haar, dB4, and Sym 8 wavelet features in various classifiers without feature selection method. Table 9 illustrates that Haar wavelet SVM with RBF kernel classifier attains a high accuracy of 77% with an error rate of 23%. In the case of the dB4 wavelet, the GMM model achieves high accuracy of 73.5% with an error rate of 26.5%. For Sym 8 wavelet, once again SVM (RBF) classifier reaches the top with high accuracy of 92.5% with an error rate of 7.5%. SVM (RBF) classifier's high accuracy demonstrates the classifier's ability to distinguish correct classes among various Features.

The article "A Framework on Performance Analysis of Mathematical Model-Based Classifiers in Detection of Epileptic Seizure from EEG Signals with Efficient Feature Selection" was published in 2022. Journal: J Healthc Eng.

Table 10 unveils the average performance measures, such as Sensitivity, Specificity, Accuracy, F1 Score, Error Rate, and G-mean for Haar, dB4, and Sym 8 wavelet features in various classifiers with PSO feature selection method. Table 10 also exemplifies that for Haar wavelet, SVM with RBF kernel classifier attains high accuracy of 87% with an error rate of 13%. In the case of the dB4 wavelet, the K-NN model achieves high accuracy of 84.5% with an error rate of 15.5%. For Sym 8 wavelet, once again SVM (RBF) classifier reaches the top with high accuracy of 90% with an error rate of 10%. Overall, high classification parameters, such as 98% accuracy, 98% F1 score, and 2% error rate are achieved in the SVM (RBF) classifier for sym 8 wavelet features with PSO feature selection.  Table 11 outlines the previous identification efforts for EEG signals. The accuracy of these efforts ranged from 73.5% to 97.3%.

The suggested approaches for linear regression, nonlinear regression, GMM, K-NN, SVM-linear, SVM-polynomial, and SVM-RBF classifiers using wavelet (Haar, dB4, sym8) and PSO features outperformed other existing approaches in epileptic seizure classification. The SVM classifier with RBF kernel in sym 8 wavelet features with the PSO feature selection method attains a higher accuracy rate of 98% with an error rate of 2%. This classifier outperforms all other classifiers.

## 6. Conclusion

Epilepsy or “seizure disorders” is a chronic disorder and is the fourth most common neurological disorder affecting people across all ages. Early diagnosis can help the patient's rehabilitation. This paper proposed the four levels of decomposition using Haar, dB4, and Sym 8 wavelet transforms for feature extraction from Bonn A and E EEG signals. The PSO technique was used to reduce the magnitude of decamped signals. Then seven classifiers were used to classify the signals as seizure and nonseizure. The SVM classifier with RBF kernel in sym 8 wavelet features with the PSO feature selection approach achieves a higher accuracy rate of 98% with a 2% error rate. This kind of classification algorithm outperforms all others. It is thereby proposed to engage further research in the direction of deep neural networks and other mathematical model-based classifiers like NBC and Random Forest.

## Figures and Tables

**Figure 1:** Schematic diagram of proposed method.

**Figure 2:** Histogram of Haar wavelet coefficient for epilepsy E-set.

**Figure 3:** Histogram of Haar wavelet coefficient for normal A-set.

**Figure 4:** Performance of MSE in number of iteration for PSO at different weights (inertia).

**Figure 5:** Normal probability plot for dB4 wavelet coefficient with PSO feature selection for epilepsy E-set.

The article "A Framework on Performance Analysis of Mathematical Model-Based Classifiers in Detection of Epileptic Seizure from EEG Signals with Efficient Feature Selection" was published in 2022. Journal: J Healthc Eng.

**Figure 6:** Normal probability plot for dB4 wavelet coefficient with PSO feature selection for normal A-set.

**Table 1:** Detailed description of the implementation environment of the study.

Dataset	Methodology		Classifiers	Software
	Feature extraction	Feature selection		
Bonn university EEG datasets (A–E). Each set input [4096 samples × 100 epochs]	Wavelet level 4 decomposition (Haar, db4, and Sym8) [256 × 100]	PSO [256 × 10]	LR, NLR, GMM, K-NN, and SVM (linear, polynomial, and RBF)	Matlab 2019a

**Table 2:** Detailed description of the EEG Bonn university datasets.

Data set	Number of epochs	Duration of epoch in seconds	Circumstances of acquisition
Set A	100	23.6	Five patients, all of them are in good health and have their eyes open
Set B	100	23.6	Five patients, all of them are in good health and have their eyes closed
Set C	100	23.6	There are five epileptics who are seizure-free
Set D	100	23.6	There are five epileptics who are seizure-free
Set E	100	23.6	Five epileptic patients with active seizure

**Table 3:** Features extracted from DWT coefficients without feature selection method.

Statistical parameters	Haar wavelet		dB4 wavelet		Sym 8 wavelet	
	A	E	A	E	A	E
Mean	6.099584	−16.7531	0.099606	−16.7328	0.02899	−16.7287
Variance	73.5206	3029.474	0.000263	3116.757	0.011726	3123.223
Skewness	1.098017	−0.01327	2.484157	−0.01253	-0.60786	−0.01397
Kurtosis	−0.71982	0.073067	5.022013	0.092693	0.117881	0.085127
Pearson correlation coefficient	0.41472	0.013761	0.005183	0.013871	0.513197	0.014305
CCA	0.534668		0.57721		0.670713	

**Table 4:** Features extracted from DWT coefficients with PSO feature selection method.

Statistical parameters	Haar wavelet		dB4 wavelet		Sym 8 wavelet	
	A	E	A	E	A	E
Mean	0.100211	39.86297	0.100678	42.9912	0.099508	42.03022
Variance	0.001501	1248.341	0.001165	2041.859	0.001941	2132.655
Skewness	−0.03815	0.753713	−0.80264	0.66277	−1.19694	0.719259
Kurtosis	12.93212	−0.94194	17.05044	−1.2422	19.47415	−1.1595
Pearson correlation coefficient	−0.01129	−0.00714	-0.00704	0.018943	0.021754	0.008678
CCA	0.13711		0.17107		0.16946	

**Table 5:** Average MSE for Haar, dB4, and Sym 8 wavelet features in various classifiers with PSO feature selection.

Wavelets	Classifiers	TP	TN	FP	FN	MSE
Haar	Linear regression	52	61	39	48	0.000212
	Nonlinear regression	64	55	45	36	0.00011
	Gaussian mixture model (GMM)	51	74	26	49	0.000231
	KNN	55	87	13	45	8.67*E* − 05
	SVM (linear)	56	53	47	44	0.0002
	SVM (polynomial)	82	80	20	18	1.23*E* − 05
	SVM (RBF)	85	89	11	15	3.48*E* − 06

dB4	Linear regression	71	81	19	29	2.12*E* − 05
	Nonlinear regression	72	77	23	28	2.23*E* − 05
	Gaussian mixture model (GMM)	55	78	22	45	0.000106
	KNN	87	82	18	13	7.44*E* − 06
	SVM (linear)	66	76	24	34	3.21*E* − 05
	SVM (polynomial)	63	66	34	37	4.9*E* − 05
	SVM (RBF)	63	93	7	37	1.96*E* − 05

Sym8	Linear regression	59	89	11	41	3.64*E* − 05
	Nonlinear regression	57	52	48	43	0.000233
	Gaussian mixture model (GMM)	64	51	49	36	0.00029
	KNN	54	52	48	46	0.000336
	SVM (linear)	53	56	44	47	0.000191
	SVM (polynomial)	55	59	41	45	0.000126
	SVM (RBF)	**90**	**90**	**10**	**10**	**1.96*E* − 06**

The article "A Framework on Performance Analysis of Mathematical Model-Based Classifiers in Detection of Epileptic Seizure from EEG Signals with Efficient Feature Selection" was published in 2022. Journal: J Healthc Eng.

**Table 6:** Confusion matrix for the seizure detection.

Confusion matrix	Class	Predicted	
		Normal	Seizure
Actual	Normal	TN	FP
	Seizure	FN	TP

**Table 7:** Values of TP, TN, FP, FN, and MSE for Haar, dB4, and Sym 8 wavelet features in various classifiers without feature selection.

Wavelets	Classifiers	TP	TN	FP	FN	MSE
Haar	Linear regression	57	66	34	43	6.48*E* − 05
	Nonlinear regression	58	57	43	42	8.38*E* − 05
	GMM	68	75	25	32	3*E* − 05
	K-NN	55	87	13	45	7.44*E* − 05
	SVM (linear)	62	72	28	38	4.16*E* − 05
	SVM (polynomial)	65	62	38	35	5.35*E* − 05
	SVM (RBF)	69	85	15	31	2.14*E* − 05

dB4	Linear regression	70	57	43	30	0.000143
	Nonlinear regression	55	66	34	45	8.29*E* − 05
	GMM	63	84	16	37	2.98*E* − 05
	K-NN	61	57	43	39	7.46*E* − 05
	SVM (linear)	72	57	43	28	5.53*E* − 05
	SVM (polynomial)	63	53	47	37	0.000199
	SVM (RBF)	53	55	45	47	0.000194

Sym8	Linear regression	54	64	36	46	0.000138
	Nonlinear regression	59	87	13	41	3.56*E* − 05
	GMM	55	73	27	45	0.000102
	K-NN	55	81	19	45	6.7*E* − 05
	SVM (linear)	71	57	43	29	5.78*E* − 05
	SVM (polynomial)	57	83	17	43	4.44*E* − 05
	SVM (RBF)	**90**	**95**	**5**	**10**	**8.89*E* − 06**

**Table 8:** Values of TP, TN, FP, FN, and MSE for Haar, dB4, and Sym 8 wavelet features in various classifiers with feature selection.

Wavelets	Classifiers	TP	TN	FP	FN	MSE
Haar	Linear regression	52	61	39	48	0.000212
	Nonlinear regression	64	55	45	36	0.00011
	GMM	51	74	26	49	0.000231
	K-NN	55	87	13	45	8.67*E* − 05
	SVM (linear)	56	53	47	44	0.0002
	SVM (polynomial)	82	80	20	18	1.23*E* − 05
	SVM (RBF)	85	89	11	15	3.48*E* − 06

dB4	Linear regression	71	81	19	29	2.12*E* − 05
	Nonlinear regression	72	77	23	28	2.23*E* − 05
	GMM	55	78	22	45	0.000106
	K-NN	87	82	18	13	7.44*E* − 06
	SVM (linear)	66	76	24	34	3.21*E* − 05
	SVM (polynomial)	63	66	34	37	4.9*E* − 05
	SVM (RBF)	63	93	7	37	1.96*E* − 05

Sym8	Linear regression	59	89	11	41	3.64*E* − 05
	Nonlinear regression	57	52	48	43	0.000233
	GMM	64	51	49	36	0.00029
	K-NN	54	52	48	46	0.000336
	SVM (linear)	53	56	44	47	0.000191
	SVM (polynomial)	55	59	41	45	0.000126
	SVM (RBF)	**98**	**98**	**2**	**2**	**1.96*E* − 06**

**Table 9:** Comparison between different classifiers with Haar, dB4, and Sym 8 wavelet features without feature selection.

Wavelets	Classifiers	Sensitivity	Specificity	Accuracy	F1 score	Error rate	G-mean
Haar	Linear regression	57	66	61.5	59.68586	38.5	61.58507
	Nonlinear regression	58	57	57.5	57.71144	42.5	57.5007
	GMM	68	75	71.5	70.46632	28.5	71.58989
	K-NN	55	87	71	65.47619	29	73.01289
	SVM (linear)	62	72	67	65.26316	33	67.14976
	SVM (polynomial)	65	62	63.5	64.03941	36.5	63.51087
	SVM (RBF)	69	85	77	75	23	77.58279

dB4	Linear regression	70	57	63.5	65.7277	36.5	63.70707
	Nonlinear regression	55	66	60.5	58.20106	39.5	60.61733
	GMM	63	84	73.5	70.39106	26.5	74.40527
	K-NN	61	57	59	59.80392	41	59.01332
	SVM (linear)	72	57	64.5	66.97674	35.5	64.79557
	SVM (polynomial)	63	53	58	60	42	58.07519
	SVM (RBF)	53	55	54	53.53535	46	54.00154

Sym8	Linear regression	54	64	59	56.84211	41	59.08392
	Nonlinear regression	59	87	73	68.60465	27	74.63016
	GMM	55	73	64	60.43956	36	64.41616
	K-NN	55	81	68	63.21839	32	69.12302
	SVM (linear)	71	57	64	66.35514	36	64.24879
	SVM (polynomial)	57	83	70	65.51724	30	71.23203
	SVM(RBF)	**90**	**95**	**92.5**	**92.30769**	**7.5**	**92.46621**

The article "A Framework on Performance Analysis of Mathematical Model-Based Classifiers in Detection of Epileptic Seizure from EEG Signals with Efficient Feature Selection" was published in 2022. Journal: J Healthc Eng.

**Table 10:** Comparison between different classifiers with Haar, dB4, and Sym 8 wavelet features with PSO feature selection.

Wavelets	Classifiers	Sensitivity	Specificity	Accuracy	F1 score	Error rate	G-mean
Haar	Linear regression	52	61	56.5	54.45026	43.5	56.55
	Nonlinear regression	64	55	59.5	61.24402	40.5	59.57134
	GMM	51	74	62.5	57.62712	37.5	63.12524
	K-NN	55	87	71	65.47619	29	73.01289
	SVM (linear)	56	53	54.5	55.17241	45.5	54.50389
	SVM (polynomial)	82	80	81	81.18812	19	81.01003
	SVM (RBF)	85	89	87	86.73469	13	87.04667

dB4	Linear regression	71	81	76	74.73684	24	76.21739
	Nonlinear regression	72	77	74.5	73.84615	25.5	74.55129
	GMM	55	78	66.5	62.14689	33.5	67.30243
	K-NN	87	82	84.5	84.87805	15.5	84.56879
	SVM (linear)	66	76	71	69.47368	29	71.18052
	SVM (polynomial)	63	66	64.5	63.95939	35.5	64.51159
	SVM (RBF)	63	93	78	74.11765	22	80.24002

Sym8	Linear regression	59	89	74	69.41176	26	75.96269
	Nonlinear regression	57	52	54.5	55.60976	45.5	54.51081
	GMM	64	51	57.5	60.0939	42.5	57.62039
	K-NN	54	52	53	53.46535	47	53.00117
	SVM (linear)	53	56	54.5	53.80711	45.5	54.50389
	SVM (polynomial)	55	59	57	56.12245	43	57.01053
	SVM (RBF)	**98**	**98**	**98**	**98**	**2**	**98**

**Table 11:** Related researches on EEG signal identification and its performance measurement constraints.

Authors	Features	Classifier	Accuracy in %
Rajaguru and Prabhakar [4]	Discrete wavelet transform (Haar, dB4, Sym8)	SVD	97.3
Murugavel and Ramakrishnan [5]	Wavelet transform with approximate entropy	SVM with ELM	96
Truong et al. [6]	EEG features	Hills algorithm	Sensitivity: 91.95 Specificity: 94.05
Manjusha and Harikumar [7]	Detrend fluctuation analysis with power spectral density	K-means clustering and KNN	Sensitivity: 90.48 Specificity: 92.85
Radüntz et al. [8]	EEG features	SVM and ANN	95.85 and 94.04
Ghaemi et al. [11]	Improved binary gravitation search algorithm with wavelet domain features	SVM	80
Kumar et al. [37]	—	Improved Elman neural network	96

In this paper	Haar wavelet features	SVM (RBF)	77
	dB4 wavelet features	GMM	73.5
	**Sym 8 wavelet features**	**SVM (RBF)**	**92.5**

In this paper	Haar wavelet + PSO features	SVM (RBF)	87
	dB4 wavelet + PSO features	K-NN	84.5
	**Sym 8 wavelet** **+** **PSO features**	**SVM (RBF)**	**98**

The article "A Framework on Performance Analysis of Mathematical Model-Based Classifiers in Detection of Epileptic Seizure from EEG Signals with Efficient Feature Selection" was published in 2022. Journal: J Healthc Eng.

## Data Availability

The data used to carry out this study can be obtained from the corresponding author upon request. The dataset of EEG can be obtained from BONN university EEG database.
